# MicroRNA-101-3p inhibits fibroblast-like synoviocyte proliferation and inflammation in rheumatoid arthritis by targeting PTGS2

**DOI:** 10.1042/BSR20191136

**Published:** 2020-01-14

**Authors:** Qiaofeng Wei, Fang Lv, Hongju Zhang, Xinfang Wang, Qin Geng, Xiuying Zhang, Tongying Li, Shujun Wang, Yajuan Wang, Yanhui Cui

**Affiliations:** 1 Department of Rheumatology, ZiBo Central Hospital, Zibo 255036, Shandong, P.R. China; 2 Department of Rheumatology, People’s Hospital of Rizhao, Rizhao 276826, Shandong, P.R. China

**Keywords:** Fibroblast-like synoviocytes, microRNA-101-3p, Prostaglandin-endoperoxide synthase 2, Rheumatoid arthritis, Synovial injury

## Abstract

**Objective:** Rheumatoid arthritis (RA) is the most frequently occurring inflammatory arthritis. The present study was performed to characterize the role of microRNA-101-3p (miR-101-3p) and prostaglandin-endoperoxide synthase 2 (PTGS2) in inflammation and biological activities of fibroblast-like synoviocytes (FLSs) in RA.

**Methods:** Initially, miR-101-3p and PTGS2 expression in RA tissues of RA patients and RA rats was detected by qRT-PCR and Western blot analysis. Rat model of type II collagen-induced arthritis (CIA) was adopted to simulate RA, followed by injection of miR-101-3p mimics or siRNA against PTGS2. Next, the apoptosis in synovial tissue and the levels of tumor necrosis factor (TNF)-α, IL-1β and IL-6 were identified. Subsequently, FLSs in RA (RA-FLSs) were isolated, after which *in vitro* experiments were conducted to analyze cell proliferation, apoptosis, migration and invasion upon treatment of up-regulated miR-101-3p and silenced PTGS2. Furthermore, the relationship of miR-101-3p and PTGS2 was determined by bioinformatics prediction and luciferase activity assay.

**Results:** We identified poorly expressed miR-101-3p and highly expressed PTGS2 in synovial tissues of RA patients and RA rats, which showed reduced synoviocyte apoptosis and enhanced inflammation. In response to miR-101-3p mimics and si-PTGS2, the RA-FLSs were observed with attenuated cell proliferation, migration and invasion, corresponding to promoted apoptosis. Down-regulation of PTGS2 could rescue the effect of inhibited miR-101-3p in synovial injury and phenotypic changes of FLS in RA rats. Notably, miR-101-3p was found to negatively regulate PTGS2.

**Conclusion:** Taken together, miR-101-3p reduces the joint swelling and arthritis index in RA rats by down-regulating PTGS2, as evidenced by inhibited FLS proliferation and inflammation.

## Introduction

Rheumatoid arthritis (RA) represents one of the most common chronic joint inflammatory diseases associated with a heavy burden for the patients and the society [1,2]. RA has been recognized to be accompanied by systemic inflammation, persistent synovitis, and autoantibodies [3]. The incidence of RA ranges from 0.5 to 1%, which decreases from urban to rural areas and from the north to the south in the northern hemisphere [4,5]. The two primary adverse outcomes caused by RA are joint damage and disability, which severely reduce the patients’ quality of life and carry a high risk of premature mortality [6,7]. Joint destruction is stimulated during the process of tissue response, when the synovial fibroblasts transform to a phenotype of aggressive inflammation and invasiveness, in addition to facilitated synovial osteoclastogenesis [8]. In RA, fibroblast-like synoviocytes (FLSs) represent the most common type of cells in cartilage junction, the activation of which stimulates joint destruction by releasing cytokines and chemokines, together with invading and migrating the joint cartilage [9]. Unfortunately, no agents have been proved to achieve effective remission in all the RA patients in spite of the advances in treatment, and the toxicities caused by the anti-rheumatic agents also inflict the patients [8]. At this point, biomarkers that can serve as therapeutic targets or indicators predicting treatment outcomes are needed. Herein, we intend to emphasize the importance to target FLSs in the current and future therapies for RA.

MicroRNAs (miRNAs) fine-tune the gene expression by enhancing the mRNA degradation or translational repression at the post-transcriptional level [10,11]. Recent evidence has reported the aberrant expression of miRNAs in RA, with involvement in T-cell mediation and promising potential as biomarkers of diagnosis, or intervention efficacy [12,13]. Accumulating miRNAs have been delineated as critical regulators of T cells, macrophages, and synovial fibroblasts during the development of RA, such as miR-155 being a significant mediator for the innate immune responses contributing to autoimmune arthritis [14,15]. Multiple studies have indicated the tumor suppressor role of microRNA-101-3p (miR-101-3p) in a variety of malignancies, like hepatocellular carcinoma [16] and bladder cancer [17]. Specifically, miR-101-3p has been suggested to attenuate the cell viability, and metastatic potential of lung carcinoma cells by targeting and inhibiting the expression of enhancer of zeste homologue 2 (EZH2) [18]. In this present study, the targeting relationship of miR-101-3p and prostaglandin-endoperoxide synthase 2 (PTGS2) was determined based on bioinformatics prediction and luciferase activity. On the other hand, PTGS2, encoding for the cyclooxygenase-2 (COX-2) enzyme, has been identified with promotive effect on tumor progression in increasing studies, and the effect may be achieved by the regulation of miRNAs [19]. For example, PTGS2 was validated as a target gene of miR-146a, which was shown to diminish PTGS2 expression by degrading the mRNA [20]. In this current study, we proposed a hypothesis that miR-101-3p may be implicated in the proliferation and inflammation of FLSs in rat models of RA, with involvement of PTGS2.

## Materials and methods

### Source of clinical synovial specimens

From January 2016 to January 2018, 42 cases of RA tissues in patients with RA diagnosed pathologically were collected. There were 30 females and 12 males, with an average age of 50.4 years. There were 32 cases of knee joint, 5 cases of hip joint, 1 case of elbow joint, 3 cases of manic joint, and 1 case of wrist joint. The normal synovial tissues in the control group came from the patients with knee meniscus injury with amputation due to trauma, anterior and posterior cruciate ligament injury, corpus liberum, and synovial fold syndrome with arthroscopic treatment.

### Experimental animals

A total of 80 specific pathogen free (SPF) female Sprague–Dawley (SD) rats (8–10 weeks old, 200–250 g) were provided by the Guangdong Experimental Animal Center. Ten rats were randomly selected as normal group and injected with equal volume of normal saline. The remaining 30 rats were used to develop RA rat model induced by type II collagen. All animals were housed under SPF conditions at 25–26°C, with relative humidity of 60–70%, 12/12 h light–dark cycle and regular supply of food and water. The litter was changed twice a week.

### Rat model simulating RA

The rat model of type II collagen-induced arthritis (CIA) was adopted to simulate the pathological changes of RA. The tail of the SD rat was injected twice with an emulsifier containing 1 mg/ml collagen, and the model was established for approximately 38 days. A certain amount of bovine type II collagen was dissolved in 10 mM glacial acetic acid to prepare solution at a concentration of 2 mg/ml, which was stirred at 4°C overnight. The completely dissolved bovine type II collagen solution was mixed with Sigma’s complete Freund’s adjuvant (or incomplete Freund’s adjuvant) in equal volume to prepare emulsifier containing collagen at a concentration of 1 mg/ml. The rats were placed in a special squirrel cage, and the tail of the rat was exposed. The experiment was carried out with the root of the rat tail fixed. The experimenter pinched the tail of the rat with his left hand and held the Hamilton micro-syringe to insert the needle at 1.5–2.0 cm from the root of the tail of the rat. And 0.1 ml emulsifier was intradermally injected. The initial inoculation was performed by using an emulsifier in which Freund’s adjuvant was completely mixed with collagen. After 3 weeks, an emulsifier in which incomplete Freund’s adjuvant and collagen were mixed was used. The emulsifier dose was the same for both injections. After 4–5 days of booster immunization, the rats developed arthritis symptoms, which are manifested by different degrees of redness and swelling of the feet. Generally, the symptoms were the heaviest at 35–38 days after the initial immunization. The CIA model rate can reach approximately 95% at 45 days after the initial immunization.

### Animal grouping

Eighty SD rats were divided into eight groups (ten per group) according to random number table, namely normal group (normal rats with regular feeding), RA group (RA rat models), mimics negative control (NC) group (RA rat models injected with miR-101-3p mimics NC through tail vein), miR-101-3p mimics group (RA rat models injected with miR-101-3p mimics through tail vein), sh-NC group (RA rat models injected with sh-NC of PTGS2 through tail vein), sh-PTGS2 group (RA rat models injected with sh-PTGS2 through tail vein), miR-101-3p inhibitors + sh-NC group (RA rat models injected with miR-101-3p inhibitors and sh-NC of PTGS2 through tail vein) and miR-101-3p inhibitors + sh-PTGS2 group (RA rat models injected with miR-101-3p inhibitors and sh-PTGS2 through tail vein). The first collagen immunization in rats was recorded as D0, and each of the oligonucleotide and the plasmid (200 μl) were injected via tail vein 1 day before the second immunization of collagen challenge (D20), and the normal group was injected with phosphate buffered saline (PBS) (200 μl). All the above oligonucleotides and plasmids were constructed and synthesized by Shanghai GenePharma Co., Ltd. (Shanghai, China).

### Joint inflammation and swelling degree score

From the 21st day after the initial immunization, the degree of joint swelling of each group was scored. The evaluation was performed twice a week, and each measurement was repeated three times. All the measurements were independently performed by the experimenter and the experimental assistant. The final result was averaged. Arthritis scoring (0–4 points) was adopted, 0 points: no arthritis; 1 point: red spots or mild swelling; 2 points: moderate swelling of joints; 3 points: severe swelling; 4 points: severe swelling and inability to bear weight. The sum of the limbs score is the arthritis index (maximum score = 16).

### Sample collection

The rats were killed 5 weeks after treatment according to grouping. The bilateral hind limbs, spleen, and serum were retained. Blood was collected by eyeball extraction and stored in a 1.5-ml Eppendorf (EP) tube, allowed to stand on ice. The blood was centrifuged at 1500 rpm to collect the supernatant (serum) in a new 1.5-ml EP tube, which was stored at −80°C. The bilateral knee joints were isolated as a whole, and the synovial tissue of left hind limb was cryopreserved. The synovial tissue of right hind limb was fixed in 10% paraformaldehyde solution, decalcified in 10% ethylene diamine tetraacetic acid (EDTA), and rinsed under running water. Then the tissue was dehydrated by the gradient ethanol, permeabilized by xylene, embedded in wax, and sliced. The embedded sections were subjected to histopathological examination.

### Hematoxylin–Eosin staining

The changes in knee joints of rats were observed by Hematoxylin–Eosin (HE) staining to analyze the degree of inflammatory cell infiltration and bone destruction. Five consecutive sections of each sample were selected, baked in a 60°C oven, dewaxed by xylene, and soaked in ethanol with decreasing concentration gradient. Next, sections were subjected to Hematoxylin staining, 1% hydrochloric acid alcohol differentiation, and 1% ammonia water treatment. The solution was counterstained by 1% Eosin, conventionally dehydrated, permeabilized, and sealed with neutral gum. Finally, the sections were observed under a microscope (LEICRAMLB2, Leica, Germany).

### Tansferase-mediated deoxyuridine triphophate-biotin nick end labeling (TUNEL) staining

Paraffin-embedded ankle sections (4 μm) and polylysine-coated slides were taken from rats in each group. The tissue slices were dewaxed with xylene, hydrated with ethanol, rinsed with PBS two times (each time for 5 min). Next, the slices were reacted with protein K working fluid at room temperature for 20 min, rinsed with PBS two times (each time for 3 min), and sealed with blocking fluid for 10 min. Subsequently, the slices were supplemented with 50 μl terminal deoxynucleotidyl transferase (TdT) reaction liquid and 50 μl streptavidin-HRP working solution and reacted at 37°C in dark for 30 min. At last, the slices were supplemented with 50 μl diaminobenzidine for development. The apoptotic nucleus was brown yellow. The number of apoptotic cells was observed and counted under a microscope.

### Enzyme-linked immunosorbent assay

Ten standard wells were set on the enzyme-labeled plate, and the standards were added in order to obtain concentrations of 30, 20, 10, 5, and 2.5 μmol/l, respectively. During the loading process, blank wells and sample wells to be tested are respectively set. Then 40 μl of the sample diluent and 10 μl of the sample to be tested (the final dilution of the sample is five times) was added to the sample well to be tested on the microplate reader. The sample was added to the bottom of the well of the microplate. After sealing with a sealing film, the plate was incubated at 37°C for 30 min. Next, 50 μl of the enzyme labeling reagent was added to each well for further incubation, and the blank well was not added. Then, the plate was added with 50 μl of developer A to each well and 50 μl of developer B to develop color for 10–15 min at 37°C without light exposure. Finally, 50 μl of the stop solution was added to each well to terminate the reaction (in this case, the blue color turned yellow). The wells were zeroed, and the absorbance of each well was measured with a wavelength of 450 nm. The measurement was carried out within 15 min after the addition of the stop solution. Taking the concentration of the standard as the abscissa and the optical density (OD) value as the ordinate, a standard curve was drawn on the coordinate paper. The corresponding concentration was identified from the standard curve according to the OD value of the sample.

### RNA extraction and quantitative reverse transcription-polymerase chain reaction (qRT-PCR)

Liquid nitrogen was added to the clinical synovial tissue or synovial tissue samples of rats in each group, which was then ground into uniform fine powder. The total RNA in the specimen was extracted by TRIzol (Invitrogen, U.S.A.), and the ratio of OD260nm/OD280nm was determined by ultraviolet spectrophotometer. The purity of the RNA was checked to ensure the OD value was 1.8–2.1. The miRNA was isolated using the PureLink FFPE Total RNA Isolation kit (Shanghai Haoran Biotechnology Co., Ltd., Shanghai, China). The miR-101-3p and other sample RNAs were reverse transcribed into cDNA using the ALL-in-one miRNA reverse transcription kit (GeneCopoeia, Rockville, MD, U.S.A.). A 2-μl aliquot of the template RNA was taken out, and then the reagent was added according to the miRNA reverse transcription system, followed by a water bath at 37°C (60 min) and 85°C (5 min). After the end of the test, the product was placed in a −80°C refrigerator for PCR. Fluorescence quantitative PCR was performed in accordance with the instructions of the SYBR® Premix Ex Taq™ II Kit (TaKaRa, Dalian, China). A 2 μl aliquot of the cDNA template frozen in the −80°C refrigerator was taken out, and the reagent was added according to the mRNA PCR system. The reaction system was shaken and mixed, and the bubbles were removed by centrifugation, and then PCR was carried out in an ABI 7500 type PCR instrument. The reaction cycle conditions were pre-denaturation at 95°C for 30 s, denaturation at 95°C for 5 s, annealing at 60°C for 34 s, extension at 72°C for 1 min, and extension at 72°C for 7 min after the last cycle, for a total of 40 cycles. The internal reference was β-actin, and all primers were designed and synthesized by Wuhan Bojie Bioengineering Co., Ltd (Wuhan, Hubei, China). The primer sequences are shown in Table 1. The 2^−ΔΔ*C*_t_^ method indicates the ratio of the expression of the target gene in the model group to that of the control group, and the formula is as follows: ΔΔ*C*_t_ = Δ*C*t_Experimental group_ − Δ*C*t_control group_ and Δ*C*_t_ = *C*t_gene of interest_ − *C*t_U6_. The threshold cycle is defined as the cycle at which the fluorescence intensity crosses over a level where the amplification enters a logarithmic growth phase. The experiment was repeated three times independently (this section also applies to cell experiments).

**Table 1:** Primer sequences for qRT-PCR

Gene	Primer sequence (5′–3′)
*miR-101-3p*	Forward: GCGGCGGTCAAGAGCAATAACG
	Reverse: ATCCAGTGCAGGGTCCGAGG
*PTGS2*	Forward: GGAGGTGGTGATAGCCGGTAT
	Reverse: TGGGTAATCCATAGAGCCCAG
*Caspase-3*	Forward: AACGTAGGCACCCACATAGG
	Reverse: GAAGAGACTGCCCCTGACAC
*Bax*	Forward: GGAGATGAACTGGATAGCAA
	Reverse: AGCCACAAAGATGGTCACT
*Bcl-2*	Forward: TACCGTCGTGACTTCGCAGAG
	Reverse: GGCAGGCTGAGCGGGTCTT
*U6*	Forward: GCTCGCTTCGGCAGCACAT
	Reverse: AAAATATGGAACGCTTCACG
*β-actin*	Forward: AAATCTGGCACCACACCTTC
	Reverse: GGGGTGTTGAAGGTCTCAAA

### Western blot analysis

A 30-g aliquot of tissue samples from each group was collected and ground to uniform fine powder at low temperature, followed by two PBS washes. After being added with protein lysis buffer, the tissue samples were centrifuged at 12000 rpm, 4°C for 20 min to collect the supernatant. Total protein concentration was measured using a bicinchoninic acid assay kit (P0012-1, Beyotime Institute of Biotechnology, Shanghai, China). Cells in logarithmic growth phase were centrifuged at 3000 rpm, 4°C for 20 min, and the supernatant was discarded. Then, cells were added with lysis buffer and protease inhibitor (Jiamay Biotech, Beijing, China), which were allowed to react on ice for 30 min. The protein supernatant was collected for protein quantification after centrifugation at 12000 rpm for 10 min. A 50-μg aliquot of protein was dissolved in 2× sodium dodecyl sulfate (SDS) loading buffer, and the sample was boiled at 100°C for 5 min. Then, each sample was transferred to a polyvinylidene difluoride membrane after 10% SDS/polyacrylamide gel electrophoresis (SDS/PAGE). Next, the membrane was blocked in 5% skim milk powder at room temperature for 1 h. Subsequently, the membrane was incubated with the anti-rabbit polyclonal antibodies PTGS, caspase-3, B-cell leukemia/lymphoma 2 (Bcl-2), and Bcl-2 assaciated X protein (Bax), all of which were from Abcam, Cambridge, MA, U.S.A. After washing three times with tris-buffered saline tween-20 (TBST), the membrane was incubated with a diluted (1:5000) horseradish peroxidase (HRP)-labeled goat anti-rabbit secondary antibody (SE134, Solarbio, Beijing, China) for 1 h. After TBST rinse, the protein bands were visualized by enhanced chemiluminescence reagent, and the images were captured and photographed. Absorbance analysis of the protein bands was performed using a gel imaging analysis system (JS series, Shanghai Dobio Biotech Co., Ltd., Shanghai, China). The relative expression of the sample protein = the average absorbance of the sample/the average absorbance of the internal reference. The relative expression of each sample protein was statistically analyzed.

### Isolation and characterization of FLSs

The synovial tissue from RA patients was collected, and the adipose tissue was removed. The synovial membrane was cut into small pieces of 1 mm^3^ under aseptic conditions, and washed with D-hanks solution. Approximately 2 volumes of 1 mg/ml collagenase I (Gibco, U.S.A.) was added to digest the synovial membrane in a 37°C incubator for 2 h. After the detachment, the synovial membrane was filtered through a nylon mesh of 70 μm pore size, centrifuged, and rinsed with PBS. The cells were resuspended in DMEM containing 10% FBS, and the medium was refreshed the next day [21] to obtain FLSs in RA (RA-FLSs). The morphology of the fibroblasts was observed. After the primary fibroblasts reached 80–90% confluence, the fibroblasts were digested with 0.25% EDTA-trypsin. When the fibroblasts showed cell contraction and increased cell space under the microscope, DMEM containing 10% FBS was added to stop the digestion. The cells were passaged at a ratio of 1:3. The primary and passage morphological characteristics and growth of the fibroblasts were observed under an inverted microscope (Nikon, Japan). The Vimentin protein specifically expressed in fibroblasts was identified by immunofluorescence. After the identification, fibroblasts in the logarithmic growth phase at 3–5 passages were adopted for the experiment.

### Fibroblast grouping and transfection

The RA-FLSs in the logarithmic growth phase were divided into seven groups: the blank group (RA-FLSs were not transfected), the mimics NC group (RA-FLSs transfected with miR-101-3p mimics NC), the miR-101-3p mimics group (RA-FLSs were transfected with miR-101-3p mimics), the sh-NC group (RA-FLSs were transfected with sh-NC of PTGS2), the sh-PTGS2 group (RA-FLSs were transfected with sh-PTGS2), the miR-101-3p inhibitors + sh-NC group (RA-FLSs were transfected with miR-101-3p inhibitors and sh-NC of PTGS2), and the miR-101-3p inhibitors + sh-PTGS2 group (RA-FLSs were transfected with miR-101-3p inhibitors and sh-PTGS2). The cells were seeded in six-well plates 24 h before transfection, and the cell confluence reached 30–50%. The cells were transfected according to the instructions of Lipofectamine 2000 (11668-019, Invitrogen, New York, CA, U.S.A.). A 5-μl aliquot of Lipofectamine 2000 was diluted with 250 μl of serum-free Opti-MEM, followed by incubation for 5 min at room temperature. And 100 pmol/l mimics NC and miR-101-3p mimics (final concentration of 50 nmol/l) were diluted by 250 μl of serum-free Opti-MEM (51985042, Gibco, Gaitherburg, MD, U.S.A.), followed by incubation for 5 min at room temperature. The above-mentioned two were mixed and incubated for 20 min at room temperature and added to the cell culture wells. After culturing for 6–8 h at 37°C, 5% CO_2_, the complete medium was refreshed and cultured for 24–48 h for the subsequent experiments.

### MTT assay

When the cell confluence of the transfected RA-FLSs reached approximately 80%, the RA-FLSs were detached with 0.25% trypsin to prepare a single cell suspension. After cell counting, 3 × 10^3^ to 6 × 10^3^ cells per well were seeded in a 96-well plate at a volume with 200 μl per well. Ten wells of each group were repeated. After incubation for a period of time, 20 μl of 5 mg/ml MTT solution (Sigma, U.S.A.) was added to each well. After incubation for 4 h in the incubator, the culture solution was discarded. Then, 150 μl of Dimethyl Sulfoxide (Sigma, U.S.A.) was added to each well, which was shaken gently for 10 min. At 24, 48, and 72 h, the OD value of each well was measured on a microplate reader at a wavelength of 490 nm. The cell viability curve was plotted with the time point as the abscissa and the OD value as the ordinate.

### Flow cytometry

Apoptosis was detected by Annexin V/propidium iodide (PI) double staining method. After 48 h of cell transfection, the cells were digested by 0.25% EDTA-free trypsin (PYG0107, Wuhan Boster Biological Technology Co., Ltd., Wuhan, Hubei, China) and collected in a flow tube, followed by centrifugation to discard the supernatant. The cells were washed three times with cold PBS, and the supernatant was discarded after centrifugation. According to the Annexin-V-FITC Apoptosis Detection Kit (K201-100, Biovision, U.S.A.), the Annexin-V-FITC/PI dye solution was formulated by Annexin-V-FITC, PI, hydroxyethyl piperazine ethanesulfonic acid (HEPES) buffer solution at a ratio of 1:2:50. Each 100 μl aliquot of the dye solution was adopted to resuspend 1 × 10^6^ cells, followed by incubation for 15 min at room temperature. A 1 ml aliquot of HEPES buffer solution was added to the cells. The cells were excited at 488 nm, and FITC fluorescence was detected using a 515 nm band-pass filter, while PI was detected using a 620 nm band-pass filter.

### Hoechst33258 staining

The coverslip was placed in a six-well plate. The cells after transfection for 24 h were inoculated into the six-well plate. When the cell confluence was approximately 50–80% the next day, 0.5 ml fixative was added to fix the cells for 10 min, followed by two PBS washes. A 0.5 ml aliquot of Hoechst 33258 solution (working concentration of 0.5 μg/ml) was adopted to stain cells for 5 min, followed by two PBS washes (3 min per wash). Next, one drop of antifade mounting medium was added on the glass slide, on which the coverslip with cells was covered. The nuclei stained blue were observed under a fluorescence microscope to analyze the cell morphology.

### Scratch test

Horizontal lines were evenly drawn on the back of the six-well plate using a marker at 0.5–1 cm intervals. Then, 3 × 10^4^ transfected cells were inoculated into the six-well plates with lines and cultured overnight. When the cell confluence reached 80–90% the next day, scratches were made with a pipette perpendicular to the horizontal line on the back. After 48 h of further culture, eight fields with scratches crossing by were randomly selected from each well to observe the movement of the cells at the scratches. The cells were photographed and sampled, and then the relative width of the scratches was identified by Motic Images Advanced 3.2 software to evaluate the cell migration ability. Each experiment was repeated at least three times.

### Transwell assay

Matrigel (Corning, U.S.A.) was dissolved overnight at 4°C, and then diluted at a ratio of 1:3 with serum-free DMEM. Next, 30 μl of the diluted Matrigel was added on to the membrane covering the upper chamber of each Transwell chamber (Corning, U.S.A.) in three separate times (15, 7.5, 7.5 μl) at a time interval of 10 min to allow Matrigel to spread evenly and cover all micropores on the bottom surface of the upper chamber. The cell suspension was inoculated into the Transwell upper chamber, with 3 × 10^4^ cells per well. Next, 0.5 ml of DMEM containing 10% FBS was added to the lower chamber of 24-well plate. After 48 h of incubation, the number of cells penetrating through Matrigel was counted under an inverted microscope, which was regarded as an indicator of cell invasive ability. Five fields of view were randomly selected for cell counting, and the number of cells was expressed by mean value. The experiment was repeated independently three times.

### Luciferase activity assay

Target genes of miR-101-3p was predicted using the biological prediction site targetscan.org. Besides, assays were performed to verify whether PTGS2 was a direct target gene of miR-101-3p. The miR-101-3p mimics and corresponding NC were co-transfected into 293 cells with luciferase reporter vector to construct pGL3-basic luciferase reporter gene vector. Meanwhile, the pGL3-PTGS2 plasmid and *Renilla* luciferase reporter gene vector pRL-TK (internal reference) were co-transfected. The transfection was conducted according to the instructions of the FuGENEHD (Roche, U.S.A.). Then, the dual luciferase activity assay was performed according to the instructions of the dual luciferase reporter assay system (Promega, U.S.A.). The *Renilla* luciferase activity pRL-TK (R value) was examined. The ratio of pGL3 firefly luciferase activity to *Renilla* luciferase activity pRL-TK (F/R) represents the relative luciferase activity of each group. The relative luciferase activity was calculated from three replicate experiments.

### Statistical analysis

The data were analyzed by SPSS 21.0 (SPSS, Inc, Chicago, IL, U.S.A.) statistical software. Kolmogorov–Smirnov test was used to determine normal distribution. The results were expressed as mean ± standard deviation. The *t* test was conducted for the comparison between two groups, and one-way analysis of variance (ANOVA) for the comparison among multiple groups. The pairwise comparison following ANOVA was carried out by the least significant difference *t* test (LSD-t). Two-sided *P*-values below 0.05 were considered significant.

## Results

### Synovial tissue of RA patients and rats exhibits poorly expressed miR-101-3p and highly expressed PTGS2

The expression of miR-101-3p and PTGS2 in RA tissues and normal tissues in 42 patients with RA was detected by qRT-PCR and Western blot analysis. The results showed that the expression level of miR-101-3p in RA tissues was significantly lower, while the expression of PTGS2 mRNA and protein was significantly higher than that in normal tissues (all *P*<0.05; Figure 1A,B).

**Figure 1:** Expression levels of miR-101-3p and PTGS2 in synovial tissue of rats in each group (**A**) qRT-PCR detection of miR-101-3p and PTGS2 expression in synovial tissue of patients with RA. (**B**) Western blot analysis detection of PTGS2 protein expression in synovial tissue of patients with RA. (**C**) Expression levels of miR-101-3p and PTGS2 in synovial tissue of RA rats. (**D**) Western blot analysis detection of PTGS2 protein expression in synovial tissue of RA rats. (**E**) Expression levels of miR-101-3p and PTGS2 in synovial tissue of RA rats with interference of miR-101-3p and PTGS2 expression. (**F**) PTGS2 protein expression in synovial tissue of RA rats with interference of miR-101-3p and PTGS2 expression. The data analysis between the two groups was compared with the *t* test. The data analysis among multiple groups was performed using one-way ANOVA, followed by pairwise comparison using LSD-*t*. *P<0.05 vs. the normal tissues. ^a^*P*<0.05 vs. the normal group; ^b^*P*<0.05 vs. the mimic-NC group; ^c^*P*<0.05 vs. the sh-NC group; ^d^*P*<0.05 vs. the miR-101-3p inhibitors + sh-NC group.

Additionally, the expression of miR-101-3p and PTGS2 in synovial tissues of normal rats and RA rats was detected by qRT-PCR and Western blot analysis. The results showed that the expression of miR-101-3p in the synovial tissues of RA group was significantly decreased, while the expression of PTGS2 mRNA and protein elevated, as compared with the normal group (all *P*<0.05) (Figure 1C,D), suggesting that miR-101-3p and PTGS2 may be involved in RA occurrence.

We further verified the altered expression of miR-101-3p and PTGS2 on the expression of miR-101-3p and PTGS2 in synovial tissues of rats by qRT-PCR and Western blot analysis, and we found that expression of miR-101-3p was increased and the expression of PTGS2 decreased in the miR-101-3p mimics group compared with the mimic-NC group (all *P*<0.05). Compared with the sh-NC group, the expression of miR-101-3p was not significantly changed in the sh-PTGS2 group (*P*>0.05), and the expression of PTGS2 was decreased (*P*<0.05). Relative to the miR-101-3p inhibitors + sh-NC group, the expression of miR-101-3p in the miR-101-3p inhibitors + sh-PTGS2 group was not significantly different (*P*>0.05), and the expression of PTGS2 was decreased (*P*<0.05; Figure 1E,F).

### Up-regulation of miR-101-3p and down-regulation of PTGS2 reduce foot swelling and arthritis score in RA rats

There was no redness in the paws of rats in the normal group. The paws in the RA group, mimic-NC group, sh-NC group, and the miR-101-3p inhibitors + sh-PTGS2 group were obviously red and swollen with abnormalities. The rats in the miR-101-3p mimics group and sh-PTGS2 group had only slight redness and no obvious deformity. The rats in the miR-101-3p inhibitors + sh-NC group had severe deformity of feet and claws. From the third week onward, the inflammation of the limbs of each group of rats was scored (Figure 2). The results showed that from the sixth week, the arthritis scores of rats in each group showed a large difference, and the arthritis score of the RA group increased compared with the normal group (*P*<0.05). The arthritis scores of rats declined in the miR-101-3p mimics group, sh-PTGS2 group and miR-101-3p inhibitors + sh-PTGS2 group versus the mimic-NC group, sh-NC group, and the miR-101-3p inhibitors + sh-NC group, respectively (all *P*<0.05).

**Figure 2:** Quantitation of arthritis scores of rats in each group The data analysis was performed using one-way ANOVA, followed by pairwise comparison using LSD-*t*. ^a^*P*<0.05 vs. the normal group; ^b^*P*<0.05 vs. the mimic-NC group; ^c^*P*<0.05 vs. the sh-NC group; ^d^*P*<0.05 vs. the miR-101-3p inhibitors + sh-NC group.

### Up-regulation of miR-101-3p and down-regulation of PTGS2 inhibit pathological damage of synovial tissues in RA rats

HE staining (Figure 3A) results showed that there was no inflammatory cell infiltration in the synovial tissue of the normal group, and no synovial hyperplasia was observed. In the RA group, mimic-NC group, sh-NC group, and the miR-101-3p inhibitors + sh-PTGS2 group, the inflammatory changes of the synovial tissue were observed, with plenty of monocytes, lymphocytes, neutrophil infiltration, and greatly proliferated FLSs. Besides, collagen fiber deposition was identified in the synovial tissue, accompanied by severe fibrosis in some cells, and obviously destroyed articular cartilage structure. The rats in the miR-101-3p mimics group and sh-PTGS2 group showed mild inflammation in synovial tissue, and a small amount of inflammatory cell infiltration. Moreover, the cells of the synovial layer were evenly arranged, without obvious hyperplasia, vasospasm formation, or obvious damage to the articular cartilage structure. In the miR-101-3p inhibitors + sh-NC group, the surface of synovial tissue in rats was rough, the synoviocytes were severely hyperplasia and disorderly arranged, and the number of synoviocytes was also increased, reaching five to ten layers or more, and a large amount of fibrous tissue hyperplasia could be seen in the lower synovial layer.

**Figure 3:** Pathological observation of synovial tissues and apoptosis of synoviocytes in each group (**A**) HE staining was used to observe the pathological condition of synovial tissue in each group (×400). (**B**) TUNEL staining was used to detect the apoptosis of rat synoviocytes (×200). (**C**) The apoptosis cells in each group. (**D**) Western blot assay was used to detect the expression of apoptosis-related proteins in the synovial tissue. The data analysis was performed using one-way ANOVA, followed by pairwise comparison using LSD-*t*. ^a^*P*<0.05 vs. the normal group; ^b^*P*<0.05 vs. the mimic-NC group; ^c^*P*<0.05 vs. the sh-NC group; ^d^*P*<0.05 vs. the miR-101-3p inhibitors + sh-NC group.

The results of TUNEL staining (Figure 3B,C) showed that there were fewer apoptotic synoviocytes in the synovial tissue of the normal group. Compared with the normal group, the number of apoptotic synoviocytes in the RA group decreased significantly (*P*<0.05). The number of apoptotic synoviocytes in the RA + mimics group was significantly increased in the miR-101-3p mimics group, sh-PTGS2 group and miR-101-3p inhibitors + sh-PTGS2 group versus the mimic-NC group, sh-NC group, and the miR-101-3p inhibitors + sh-NC group, respectively (all *P*<0.05).

The results of Western blot assay (Figure 3D) showed that the expression of caspase-3 and Bax in the synovial tissue of the RA group were significantly declined, relative to the normal group, accompanied by elevated expression of Bcl-2 (all *P*<0.05). The expression of caspase-3 and Bax in the synovial tissue of rats was significantly higher while expression of Bcl-2 was lower in the miR-101-3p mimics group, sh-PTGS2 group, and miR-101-3p inhibitors + sh-PTGS2 group versus the mimic-NC group, sh-NC group, and the miR-101-3p inhibitors + sh-NC group, respectively (all *P*<0.05).

### Up-regulation of miR-101-3p and down-regulation of PTGS2 inhibit inflammatory injury in RA rats

The results of qRT-PCR and Enzyme-linked immunosorbent assay (ELISA) (Figure 4A,B) displayed that the mRNA expression of IL-1β, IL-6, and tumor necrosis factor (TNF)-α in the synovial tissues and their contents in serum of the RA group were significantly increased, when compared with the normal group (all *P*<0.05). Versus the mimic-NC group, sh-NC group and the miR-101-3p inhibitors + sh-NC group, the synovial tissue of the miR-101-3p mimics group, sh-PTGS2 group, and miR-101-3p inhibitors + sh-PTGS2 group led to reduced mRNA expression of IL-1β, IL-6, and TNF-α in the synovial tissues and their contents in serum (all *P*<0.05). The results indicated that overexpression of miR-101-3p and down-regulation of PTGS2 attenuated inflammatory injury in RA rats.

**Figure 4:** Quantitation of the mRNA expression of inflammatory factors in synovial tissue and their serum levels of rats in each group (**A**) qRT-PCR was used to detect the mRNA expression of inflammatory factors in rat synovial tissue. (**B**) ELISA was used to detect the serum levels of inflammatory factors in rats. *n*=5. The data analysis was performed using one-way ANOVA, followed by pairwise comparison using LSD-*t*. ^a^*P*<0.05 vs. the normal group; ^b^*P*<0.05 vs. the mimic-NC group; ^c^*P*<0.05 vs. the sh-NC group; ^d^*P*<0.05 vs. the miR-101-3p inhibitors + sh-NC group.

### Morphological observation and identification of FLSs

The primary FLSs of RA rats were isolated and cultured by tissue block culture method. After 1–2 days, the FLSs of long fusiform shape migrated from the edge of the tissue block and gradually increased radially. After 1 week of culture, the morphology of the cells was observed by an inverted microscope (Figure 5A). The morphology of the cultured cells was conformed to show the morphological characteristics of fibroblasts, which were spindle-shaped, star-shaped, or fusiform-shaped, and some of them were polygonal. The nucleus, with a clear border and oval shape, was located in the middle of the cell, and the nucleolus was clear. When cultured to the third passage, the dendritic cells, endothelial cells, adipocytes, and vascular endothelial cells with typical morphological characteristics disappeared under the microscope, and no suspended cells were observed. Vimentin immunocytochemical staining results (Figure 5B) demonstrated that the third passage of FLSs were Vimentin positive, and a large number of brownish yellow particles were seen in the cytoplasm.

**Figure 5:** Morphological observation and immunocytochemical identification of FLSs (**A**) Morphology of third-passage FLSs of RA (400×). (**B**) Vimentin immunocytochemical staining of FLSs (200×).

### Up-regulation of miR-101-3p and down-regulation of PTGS2 inhibit proliferation of RA-FLSs

The MTT assay was used to detect the effect of miR-101-3p and PTGS2 on the proliferation of RA-FLSs (Figure 6). The OD values of RA-FLSs in each group were not significantly different at 24 h (*P*>0.05), suggesting that miR-101-3p had no significant effect on RA-FLS proliferation at 24 h. After culture of RA-FLS for 48 and 72 h, there was no significant difference in cell proliferation in the mimics-NC group compared with the blank group (*P*>0.05). The miR-101-3p mimics group, sh-PTGS2 group, and miR-101-3p inhibitors + sh-PTGS2 group displayed decreased cell proliferation (all *P*<0.05) relative to the mimic-NC group, sh-NC group, and the miR-101-3p inhibitors + sh-NC group, respectively. The aforementioned results indicate that miR-101-3p and silenced PTGS2 inhibit RA-FLS proliferation.

**Figure 6:** MTT assay verifies the effect of miR-101-3p and PTGS2 on the proliferation of RA-FLSs after transfection The data analysis was performed using one-way ANOVA, followed by pairwise comparison using LSD-*t*. The experiment was repeated three times. ^a^*P*<0.05 vs. the mimic-NC group; ^b^*P*<0.05 vs. the sh-NC group; ^c^*P*<0.05 vs. the miR-101-3p inhibitors + sh-NC group.

### Up-regulation of miR-101-3p and down-regulation of PTGS2 enhance apoptosis of RA-FLSs

The results of Annexin V-FITC/PI double staining assay are shown in Figure 7A. No significant difference in apoptosis rate was observed between the blank group and the mimics-NC group (*P*>0.05). The miR-101-3p mimics group, sh-PTGS2 group, and miR-101-3p inhibitors + sh-PTGS2 group exhibited promoted cell apoptosis (all *P*<0.05) relative to the mimic-NC group, sh-NC group and the miR-101-3p inhibitors + sh-NC group, respectively. The Hoechst 33258 staining results are shown in Figure 7B. There was no obvious morphological changes of apoptosis in the mimic-NC group, sh-NC group and the miR-101-3p inhibitors + sh-PTGS2 group. However, chromatin aggregation, DNA fragmentation, cell pyknosis, nucleus collapse, as well as the sign that nuclear fragments were completely surrounded by nuclear membrane into a spherical shape could be observed in the miR-101-3p mimics group and sh-PTGS2 group. Besides, the highlight caused by chromatin shrinkage was observed, and typical apoptotic bodies were formed. No apoptotic phenomenon was witnessed in the miR-101-3p inhibitors + sh-NC group.

**Figure 7:** Annexin V-FITC/PI double staining and Hoechst 33258 staining of apoptosis detection in RA-FLSs after transfection (**A**) Flow cytometric detection of RA-FLS apoptosis in each group. (**B**) Hoechst 33258 staining for RA-FLS apoptosis in each group. The data analysis was performed using one-way ANOVA, followed by pairwise comparison using LSD-*t*. The experiment was repeated three times. ^a^*P*<0.05 vs. the mimic-NC group; ^b^*P*<0.05 vs. the sh-NC group; ^c^*P*<0.05 vs. the miR-101-3p inhibitors + sh-NC group.

### Up-regulation of miR-101-3p and down-regulation of PTGS2 inhibit migration and invasion of RA-FLSs

The results of the scratch test and Transwell invasion assay (Figure 8A,B) showed that relative to the mimic-NC group, sh-NC group and the miR-101-3p inhibitors + sh-NC group, the migration and invasion ability was significantly suppressed in the miR-101-3p mimics group, sh-PTGS2 group and miR-101-3p inhibitors + sh-PTGS2 group, respectively (all *P*<0.05).

**Figure 8:** Scratch test and Transwell invasion assay indicate the roles of miR-101-3p and PTGS2 in cell migration and invasion ability of RA-FLSs after transfection (**A,B**) Representative images (×100) and quantitation of scratch healing rate of each group detected by scratch test. (**C,D**) Representative images (×200) and quantitation of the number of invasive cells of each group detected by Transwell invasion assay. The data analysis was performed using one-way ANOVA, followed by pairwise comparison using LSD-*t*. The experiment was repeated three times. ^a^*P*<0.05 vs. the mimic-NC group; ^b^*P*<0.05 vs. the sh-NC group; ^c^*P*<0.05 vs. the miR-101-3p inhibitors + sh-NC group.

### MiR-101-3p targets and negatively regulates PTGS2

Based on the results of qRT-PCR and Western blot assay (Figure 9A,B), we found that expression of miR-101-3p in RA-FLSs was increased and the expression of PTGS2 decreased in the miR-101-3p mimics group compared with the mimic-NC group (all *P*<0.05). Compared with the sh-NC group, the expression of miR-101-3p in RA-FLSs was not significantly changed in the sh-PTGS2 group (*P*>0.05), and the expression of PTGS2 was decreased (*P*<0.05). Relative to the miR-101-3p inhibitors + sh-NC group, the expression of miR-101-3p in RA-FLSs in the miR-101-3p inhibitors + sh-PTGS2 group was not significantly different (*P*>0.05), and the expression of PTGS2 was decreased (*P*<0.05).

**Figure 9:** Targeting relationship of miR-101-3p and PTGS2 determined based on bioinformatics prediction and luciferase activity assay (**A**) qRT-PCR was used to detect the expression of miR-101-3p and PTGS2 in each group. (**B**) Western blot assay was used to detect the protein expression of PTGS2 in each group. (**C**) Binding sites between miR-101-3p and PTGS2 were predicted by bioinformatics analysis. (**D**) Dual luciferase reporter assay analysis. The data analysis was performed using one-way ANOVA, followed by pairwise comparison using LSD-*t*. The experiment was repeated three times. ^a^*P*<0.05 vs. the mimic-NC group; ^b^*P*<0.05 vs. the sh-NC group; ^c^*P*<0.05 vs. the miR-101-3p inhibitors + sh-NC group.

Through the bioinformatics analysis of targetscan.org website, miR-101-3p was predicted to directly bind to the sequences of PTGS2 3′-UTR (Figure 9C,D). Compared with the co-transfection group of PTGS2-wt and miR-101-3p NC, luciferase activity was significantly lower in the co-transfection group of PTGS2-wt and miR-101-3p mimic (*P*<0.05). Compared with the co-transfection group of PTGS2-mut and miR-101-3p NC, there was no significant difference from the co-transfection group of PTGS2-mut and miR-101-3p mimic (*P*>0.05). This indicates regulatory targeting relationship between miR-101-3p and the 3′-UTR of PTGS2.

## Discussion

RA represents a chronic inflammatory polyarthritis, which commonly progresses to joint destruction and even disability [22]. It is important to note that the invasiveness of FLSs has been linked with the articular damage in RA [23], which plays a key role in forming the synovial pannus and generating pro-inflammatory cytokines [24]. At this point, a novel potential to develop therapeutic targets aimed at improving remission could be identified with better understanding of the biomarkers mediating invasiveness of FLSs in RA. The findings of the presents study provided evidence demonstrating the inhibitory role of miR-101-3p in the proliferation of FLSs and inflammation in rat models of RA by targeting PTGS2.

In the synovial tissue of RA rats, we revealed the poorly expressed miR-101-3p and highly expressed PTGS2, which was found to reduce joint swelling and arthritis score. It has been well established that the joint swelling in RA directly reflects the inflammation in synovial tissues following immune activation, with leukocyte infiltration into the normal synovial compartment [1]. Besides, up-regulation of miR-101-3p and down-regulation of PTGS2 were revealed to relieve pathological damage of synovial tissues, as well as facilitated apoptotic synoviocytes corresponding to increased caspase-3 and Bax and decreased Bcl-2. As the study of Sabeh et al. [25] stated, the expansion of the synoviocytes could result in the destructive remodeling of joints in addition to connective tissues. Besides, Lee et al. [26] have provided data indicating that the responsiveness of the synoviocytes to apoptosis induced by methotrexate could act as an indicator predicting the sensitivity of patients to the treatment of methotrexate. Therefore, when the miR-101-3p mimics and si-PTGS2 caused significant declines in the apoptotic synoviocytes, the pathological damage of synovial tissues should be alleviated.

Furthermore, the treatment of miR-101-3p mimics and si-PTGS2 acted to reduce inflammation in RA rats by lowering serum levels of IL-1β, IL-6, and TNF-α, coupled with their mRNA expression. Based on the evolving concepts of RA proposed by Firestein et al. [27], the personalized therapeutic strategies can be focused on diminishing synovial inflammation as well as joint destruction in RA. The imbalance between the cytokine production of pro-inflammatory and anti-inflammatory properties in the rheumatoid joints has been highlighted to induce autoimmunity and chronic inflammation, thus leading to joint damage [28]. The inflammatory milieu in the process of RA is modulated by a regulatory network of cytokines and chemokines, among which TNF, IL-6 are especially critical [29]. Mechanistically, a previous *in vitro* study focusing on inflammation-promoted lung tumorigenesis suggested that IL-1β down-regulates the expression of tumor suppressor miR-101 via the COX2-hypoxia-inducible factor (HIF)1α pathway by targeting Lin28B [30]. Besides, the inflammatory injury in the lung could be achieved in response to up-regulation of miR-101 and inhibition of IL-1β [31]. The effect of IL-1β witnessed an increased production of PTGS2 and all cytokines in osteoarthritic synovial fluid [32]. Moreover, the increased level of IL-6 and the IL-6 receptor is linked with the activation of osteoclasts, osteoclast differentiation, in addition to the generation of acute phase reactants, which have been reported to associate with synovitis and joint destruction in RA [8]. Accordingly, when the IL-1β, IL-6, and TNF-α were curtailed by miR-101-3p mimics and si-PTGS2 in RA rats, the inflammatory injury could be combated.

It is essential to note that up-regulation of miR-101-3p could repress the robust expression of PTGS2 in synovial tissue of RA rats. In addition, miR-101-3p was validated to target and negatively regulate PTGS2 expression on the basis of based on bioinformatics prediction and luciferase activity assay. Multiple studies have established that miRNAs target mRNAs for degradation from an epigenetic aspect, thus controlling cellular responses [33,34]. The role of miR-101 in controlling cell activities has been demonstrated to associate with target genes. For instance, the repression of miR-101 in the productive herpes simplex virus type 1 (HSV-1) replication in HSV-1-infected HeLa cells was achieved by targeting the *ATP5B* gene [35]. Additionally, the tumor suppressor role of miR-101-3p in cancers has also been identified by targeting and negatively regulating the target gene, such as in gastric carcinoma by targeting SFR and in hepatocellular carcinoma by targeting Rab5a [36,37]. At the same time, the promotion role of PTGS2 in breast cancer could be attenuated by up-regulation of miR-26b by regulating cell proliferation [19].

More importantly, the findings revealed that up-regulation of miR-101-3p and down-regulation of PTGS2 led to diminished proliferation, migration, and invasion of FLSs, coupled with accelerated apoptosis. Accumulating studies have proved the association of FLSs with the pathogenesis of RA through producing effector molecules, thereby expediting the inflammation and joint damage [38,39]. Resistance to apoptosis of FLSs in RA is common in the inflamed joint as a prominent characteristic [9]. Additionally, up-regulation of miR-101 caused pronounced declines in the migration and invasion of esophageal squamous cell carcinoma cells, coupled with enhanced cell apoptosis [40]. A prior study has demonstrated that PTGS2 influences carcinogenesis via modulation of angiogenesis, apoptosis, as well as cytokine expression [41]. Another study has suggested that PTGS2 (COX-2) inhibitors may restrict hypopharyngeal cancer cells proliferation through enhancement of G_1_ growth arrest [42]. Since the growth and migration of FLSs were inhibited by miR-101-3p through targeting PTGS2, the development of RA could be curtailed.

The conducted study has provided evidence suggesting that up-regulation of miR-101-3p and down-regulation of PTGS2 alleviated the inflammation and joint damage in RA, accompanied by diminished proliferation, migration, and invasion, and resistance to apoptosis of FLSs. It would be of interest to investigate further the expression of miR-101-3p during different phases of RA, and this will be the subject of future experiments. In addition, miRNA-based therapeutics may become an approach of personalized therapy in the future for enhancing therapeutic outcome, not only against RA, but also in other inflammatory diseases.

## Abbreviations

ANOVA: analysis of variance
Bax: Bcl-2 assaciated X protein
Bcl-2: B-cell leukemia/lymphoma 2
CIA: collagen-induced arthritis
COX-2: cyclooxygenase-2
EDTA: ethylene diamine tetraacetic acid
EP: Eppendorf
EZH2: enhancer of zeste homologue 2
FLS: fibroblast-like synoviocyte
HE: Hematoxylin–Eosin
HEPES: hydroxyethyl piperazine ethanesulfonic acid
HIF: hypoxia-inducible factor
HRP: horseradish peroxidase
HSV-1: herpes simplex virus type 1
LSD-t: least significant difference *t* test
miRNA: microRNA
miR-101-3p: microRNA-101-3p
NC: negative control
OD: optical density
PBS: phosphate buffered saline
PI: propidium iodide
PTGS2: prostaglandin-endoperoxide synthase 2
RA: rheumatoid arthritis
RA-FLS: FLS in RA
SD: Sprague–Dawley
SPF: specific pathogen free
TBST: tris-buffered saline tweeen-20
TdT: terminal deoxynucleotidyl transferase
TNF: tumor necrosis factor
TUNEL: transferase-mediated deoxyuridine triphophate-biotin nick end labeling
